This article has been retracted.

# Antiviral Activity of *Plantago asiatica* Polysaccharide against Pseudorabies Virus *In Vitro*

**DOI:** 10.1155/2022/3570475

**Published:** 2022-01-20

**Authors:** Changchao Huan, Wei Zhang, Yao Xu, Bo Ni, Song Gao

**Affiliations:** ^1^Institutes of Agricultural Science and Technology Development, College of Veterinary Medicine, Yangzhou University, Yangzhou, 225009 Jiangsu, China; ^2^Jiangsu Co-innovation Center for Prevention and Control of Important Animal Infectious Diseases and Zoonoses, Yangzhou, 225009 Jiangsu, China; ^3^Key Laboratory of Avian Bioproduct Development, Ministry of Agriculture and Rural Affairs, Yangzhou, 225009 Jiangsu, China; ^4^China Animal Health and Epidemiology Center, Qingdao, China; ^5^Institutes of Agricultural Science and Technology Development, Yangzhou University, China

## Abstract

Pseudorabies (PR) is an acute infectious disease of various domestic animals and wild animals caused by pseudorabies virus (PRV). It is mainly characterized by fever, itching, encephalomyelitis, and respiratory and neurological disorders. *Plantago asiatica* polysaccharide (PLP), extracted from the whole plant of *Plantago asiatica* L., showed immunomodulatory and antioxidation effects, but the antiviral activity had not been reported. In this study, the inhibitory effect of PLP on PRV infection was studied. Our study first revealed that PLP could inhibit PRV infection in a dose-dependent manner. By adding PLP at different stages of the virus's life cycle, we revealed that PLP could reduce the attachment and penetration of PRV into PK15 cells. The inhibition of PRV attachment was better than inhibition of PRV penetration. However, PLP did not affect PRV replication and inactivation. In addition, PLP decreased the intracellular ROS levels in infected cells significantly, and ROS scavenger NAC decreased PRV infection. Therefore, our study provided preliminary data of anti-PRV activity of PLP, which was established to be a novel anti-PRV infection agent.

## 1. Introduction

Pseudorabies (PR) represents the acute infectious disorder in domestic and wild animals resulting from pseudorabies virus (PRV). It is mainly characterized by fever, itching, encephalomyelitis, and respiratory and neurological disorders [1, 2]. It spreads mainly through direct contact or airborne droplets containing the virus [3]. PR first occurred in 1813, and the infected cattle showed extreme itching symptoms, similar to rabies; therefore, it was called “pseudorabies” [4]. PR was transmitted from cattle to pigs after the 1970s [5]. Since 2011, the new PRV variant has led to an epidemic in the pig immunization field in China [6, 7]. Due to the poor protective effect of the classical vaccine, it caused huge losses and resulted in great resistance to the purification of pseudorabies [8]. PRV was recently isolated from a patient with acute human encephalitis [9]. Therefore, to reduce the economic loss caused by PRV, developing novel antiviral agents for inhibiting PRV infection is of great urgency.

Extracts from the Chinese herbal medicines, particularly the corresponding polysaccharides, have shown antiviral activity. *Radix isatidis* polysaccharide [10], *Platycodon grandiflorus* polysaccharides [11], and kumazasa extract [12] were verified to inhibit PRV infection. The efficacy of such polysaccharides is associated with PRV replication inhibition, the direct killing of PRV, and downregulation of PRV-induced autophagy. These studies offer the foundation to apply polysaccharides in a clinic.

*Plantago asiatica* L., as a Plantaginaceae family member, can be easily cultivated and is widely distributed in eastern Asia [13]. *Plantago asiatica* L. is used to be a folk medicine since ancient times [14]. As revealed by pharmacological articles, plantain possesses antiulcer, antidiarrheal, anti-inflammatory, analgesic, antioxidant, anticancer, and antiviral activities [15, 16]. Phytochemical studies showed that the main chemical components of *Plantago asiatica* L. are lipids, polysaccharides, iridoid glycosides, alkaloids, flavonoids, and caffeic acid derivatives [13]. Polysaccharides in *Plantago asiatica* L. (PLP) leaves have several biological activities. PLP displays the effect of immunomodulation through the stimulation of pro-inflammatory cytokine generation [17]. PLP is suggested to promote the production of TNF-*α* and nitric oxide (NO) via macrophage activation [18]. However, the antiviral activity of PLP has not been reported, and PK15 cells are generally used in *in vitro* PRV research [19]. Thus, we studied PLP's role in resisting PRV within PK15 cells.

Therefore, our work evaluated the antiviral activity of PLP against PRV *in vitro* and showed that PLP plays an anti-PRV role by mainly inhibiting the attachment and penetration of PRV and decreasing ROS production. Our findings can offer guidance for PLP application, especially in clinical applications as antiviral medicines.

## 2. Materials and Methods

### 2.1. Cell Culture and Virus Preservation

We cultivated cells at 37°C and 5% CO_2_ conditions and cultivated PK15 cells within DMEM containing 5% fetal bovine serum (FBS), whereas Vero cells within DMEM contained 6% FBS. All the viruses were preserved at –80°C. We isolated PRV XJ5 strain in our laboratory.

### 2.2. Chemicals, Reagent, and Antibodies

*Plantago asiatica* polysaccharides (≥98% (uv)) obtained from Yangling Ciyuan Biotechnology Co., Ltd., China was diluted with PBS to 50 mg/mL, followed by preservation at –20°C. The citric acid solution was constituted by citric acid (40 mM), NaCl (135 mM), and KCl (10 mM), and pH was adjusted to 3.0. DAPI was provided by Beyotime Biotechnology (Shanghai, China). In addition, the PRV gB antibody and the PRV-positive serum were prepared and preserved at our laboratory. We obtained a *β*-actin antibody in Beijing genetically modified Biotechnology Co., Ltd. (Beijing, China), and the goat anti-porcine IgG antibody labeled with FITC was purchased from Sigma-Aldrich (St. Louis, MO).

### 2.3. Infectivity Assay

PK15 cells (5 × 10^5^/well) were laid in a six-well plate and cultivated under 5% CO_2_ and 37°C conditions until they grew to a density of 70–80%. After discarding the original culture medium, we rinsed cells thrice using PBS. We cultured PK15 cells within DMEM that contained various concentrations of PLP (100, 200, 400, and 600 *μ*g/mL) for a 1 h period at 37°C. After that, we inoculated PRV XJ5 (multiplicities of infection (MOI) = 0.1) into cells. After infection for 1 h, we discarded virus solution and rinsed cells thrice using PBS. Then, we cultured cells in 2% DMEM containing PLP (100, 200, 400, and 600 *μ*g/mL) at 37°C. After 24 h postinfection (hpi), we harvested cells to detect viral proteins in cells through WB analysis and collected supernatants for detecting virus titers through TCID_50_.

We pretreated PK15 cells for a 1 h period with PLP (600 *μ*g/mL), followed by another 1 h PRV XJ5 (MOI = 0.1) infection. Then, we rinsed cells thrice using PBS, followed by the culture in 2% DMEM that contained PLP (600 *μ*g/mL). At 2, 4, 8, 12, and 24 hpi, we measured gB protein expression through WB assay.

PK15 cells were pretreated with PLP (400 and 600 *μ*g/mL) and infected with different MOI of PRV XJ5 (MOI = 0.1, 0.5, 1, and 2) for a 1 h period. Then, we rinsed cells thrice using PBS, followed by the culture within 2% DMEM containing PLP (400 and 600 *μ*g/mL). At 24 hpi, we harvested cells for detecting gB protein level by WB assay.

### 2.4. Pretreatment Assay

PK15 cells were pretreated with corresponding PLP concentrations (100, 200, 400, and 600 *μ*g/mL) for a 1 h period at 37°C. After washing thrice using PBS, cells were inoculated with PRV XJ5 (MOI = 0.1) for a 1 h period. Cell supernatants were eliminated, followed by cell rinsing thrice by PBS. Finally, we incubated PK15 cells at 37°C within 2% DMEM. At 24 hpi, we harvested cells for detecting the gB protein level through WB analysis.

### 2.5. Attachment and Penetration Assay

We rinsed PK15 cells thrice using prechilled PBS, followed by infection using PRV XJ5 (MOI = 0.1) in DMEM containing PLP (100, 200, 400, and 600 *μ*g/mL) for a 1 h period under 4°C without pretreatment. After rinsing cells using cold PBS thrice, cells were cultured with 2% DMEM with PLP (100, 200, 400, and 600 *μ*g/mL) under 37°C. At 1 h later, we discarded cell supernatants. The citric acid solution and PBS removed the uninternalized virus particle, followed by a culture of infected cells within 2% DMEM without PLP. Cells were collected at 24 hpi to detect viral protein levels within cells through the WB assay. Then, we collected cell supernatants for detecting virus titers through TCID_50_.

### 2.6. Attachment Assay

We rinsed PK15 cells thrice using prechilled PBS, followed by PRV XJ5 (MOI = 0.1) infection with PLP (100, 200, 400, and 600 *μ*g/mL) at 4°C for a 1 h period. After washing thrice using cold PBS, we kept cells with 2% DMEM without PLP for 1 h at 37°C. We harvested cells at 24 hpi, to detect viral protein levels in cells through WB, and we collected cell supernatants for detecting virus titers through TCID_50_.

### 2.7. Penetration Assay

We infected PK15 cells by PRV XJ5 (MOI = 0.1) for a 1 h period at 4°C with PLP. The cell supernatant was discarded, followed by a culture with 2% DMEM containing PLP (100, 200, 400, and 600 *μ*g/mL) for a 1 h period under 37°C. We eliminated uninternalized virus particles through a citric acid solution and PBS and cultivated those infected cells within 2% DMEM without PLP. Cells and the supernatant were collected at 24 hpi to measure the intracellular viral proteins and virus titer by western blot or TCID_50_.

### 2.8. Replication

We infected PK15 cells by PRV XJ5 (MOI = 0.1) without PLP for 1 h and washed them with PBS thrice. Thereafter, we cultured cells with 2% DMEM with PLP (100, 200, 400, and 600 *μ*g/mL) at 37°C. We harvested cells at 4 and 6 hpi for detecting viral gB protein level and viral DNA copy numbers.

### 2.9. Direct Inactivation Effects on PRV

PRV XJ5 (MOI = 0.1) was incubated with PLP (100, 200, 400, and 600 *μ*g/mL) for a 1 h period at 37°C, followed by inoculation of pretreatment virus to Vero cell to measure the virus titer by TCID_50_.

### 2.10. Intracellular ROS Assay

PK15 cells were pretreated with PLP (600 *μ*g/mL) at 37°C for a 1 h period, followed by infection by PRV XJ5 (MOI = 0.1). After 1 h, we cultivated cells in 2% DMEM using PLP (600 *μ*g/mL). At 24 hpi, after rinsing cells by PBS thrice, we incubated cells using 10 mM 2′, 7′-dichlorofluorescein diacetate (DCFH-DA) probe for a 30 min period at 37°C. We eliminated extra probes, and cells were resuscitated with PBS. Flow cytometry was conducted to measure the total fluorescence intensity of >10,000 cells in each sample.

### 2.11. Western Blotting

The cells collected were lysed with cell lysis buffer. The cell lysate protein and 5× SDS-PAGE sample loading buffer (4 : 1) were boiled in a metal bath at 96°C for 15 min. The proteins isolated through 12% SDS-PAGE were transferred from the gel onto nitrocellulose (NC) membrane. Later, we blocked the NC membrane using 3% nonfat powdered milk in PBST at ambient temperature for a 2 h period, followed by overnight incubation with the primary antibody under 4°C, and then washed thrice with PBST. NC membrane was incubated in HRP-conjugated goat anti-mouse antibody for 2 h at ambient temperature. The Super ECL Reagent Solution kit (Shanghai share Biotechnology, China) was employed to analyze immune complex band results.

### 2.12. Indirect Immunofluorescence Assay (IFA)

We fixed cells using the 4% paraformaldehyde (PFA) at 37°C for a 30 min period, followed by 10 min incubation using 0.1% Triton X-100 and overnight sealing using 5% BSA at 4°C. After washing by PBS thrice, we cultured cells using PRV-positive porcine serum for a 1 h period under 37°C and then using FITC-labeled goat anti-porcine IgG antibody for a 30 min period at 37°C. Finally, we stained cells for a 7 min period using DAPI, followed by observation using a fluorescence microscope.

### 2.13. qRT-PCR

We conducted qRT-PCR according to the previous description [20]. In brief, viral DNA was isolated, followed by assessment of gene levels with specific primers: gB94, 5′-ACAAGTTCAAGGCCCACATCTAC-3′ (forward), gB94, 5′-GTCCGTGAAGCGGTTCGTGAT-3′ (reverse).

### 2.14. Virus Titer Assays

The virus titer was evaluated by TCID_50_, as performed as the previous description [20].

### 2.15. Statistical Analysis

The results were displayed in the form of mean ± SD and examined using GraphPad Prism software (GraphPad Software, San Diego, CA), and all experiments were repeated independently thrice. One-way ANOVA, as well as Duncan's multiple range test, was utilized to analyze differences between groups. ^∗^*P* < 0.05, ^∗∗^*P* < 0.01 stood for significant difference.

## 3. Results

### 3.1. PLP Inhibits PRV Infection within PK15 Cells

For measuring PLP's antiviral activity against PRV infection, we treated PK15 cells for a 1 h period with PLP at diverse doses. Thereafter, we infected cells by PRV XJ5 (MOI = 0.1) for a 1 h period with PLP and rinsed them three times using PBS. Afterwards, we cultivated cells with 2% DMEM that contained PLP (100, 200, 400, and 600 *μ*g/mL) at 37°C. At 12 and 24 hpi, the cytopathic effect (CPE) caused by PRV infection was observed using a microscope.  Figure 1(a) shows that PLP could reduce CPE in PK15 cells, suggesting that PLP can inhibit PRV infection. The western blot results further confirmed PRV gB protein expression was reduced significantly at PLP concentrations of 400 and 600 *μ*g/mL (Figure 1(b)). Furthermore, the virus titer in the cell supernatant was evaluated. The results showed that PLP reduced virion production dose dependently (Figure 1(c)). Additionally, based on IFA results, the number of infected cells decreased with the increase of PLP concentration (Figure 1(d)). According to the above findings, PLP inhibited PRV infection within PK15 cells.

For better investigating PLP's antiviral activity in PRV, we infected PK15 cells by PRV XJ5 (MOI = 0.1) with PLP (600 *μ*g/mL), cells were collected at 2, 4, 8, 12, and 24 hpi. WB results indicated that PLP could inhibit PRV infection effectively (Figure 2(a)). Furthermore, PK15 cells in the presence of PLP (400 and 600 *μ*g/mL) were subjected to PRV XJ5 infection at MOI (0.1, 0.5, 1, and 2). According to WB assay at 24 hpi, PLP inhibited different MOI PRV infections, indicating the highest antiviral activity at the decreased MOI (Figure 2(b)).

### 3.2. PLP Inhibits PRV Attachment and Penetration into PK15 Cells

To explore the antiviral effect of PLP in various PRV life cycle stages, we pretreated PK15 cells using different concentrations of PLP (100, 200, 400, and 600 *μ*g/mL) followed by 24 h infection by PRV XJ5 (MOI = 0.1) without PLP. As revealed by WB assay, PRV gB protein level was downregulated (Figure 3(a)), suggesting that pretreatment of cells affected the virus infectivity.

For investigating PLP's role in virus attachment and penetration, we infected PK15 cells for a 1 h period by PRV XJ5 (MOI = 0.1) at 4°C that contained different concentrations of PLP (100, 200, 400, and 600 *μ*g/mL). After rinsing by prechilled PBS thrice, we incubated cells by PLP for a 1 h period under 37°C and rinsed thrice by the citric acid solution and PBS for removing those noninternalized virus particles and maintained in 2% DMEM. We harvested cells at 24 hpi for detecting intracellular viral proteins using western blot. The results showed that the protein level of PRV gB reduced, especially with 400 and 600 *μ*g/mL PLP (Figure 3(b)). The supernatant was collected to measure viral titers, which revealed that PRV titer decreased dose dependently (Figure 3(c)). Besides, according to IFA assay, PLP decreased numbers of infected cells (Figure 3(d)). These results confirm that PLP inhibited PRV attachment and penetration into PK15 cells.

### 3.3. PLP Inhibits PRV Attachment to PK15 Cells

To clarify whether PLP could inhibit PRV attachment onto PK15 cells, we infected cells by PRV XJ5 (MOI = 0.1) in DMEM containing PLP (100, 200, 400, and 600 *μ*g/mL) for a 1 h period at 4°C and rinsed them thrice using prechilled PBS. Then, we cultivated cells with 2% DMEM without PLP under 37°C. At 24 hpi, the PRV gB protein expression was measured through WB. As a result, PRV gB protein decreased at PLP concentrations of 400 and 600 *μ*g/mL (Figure 4(a)). The supernatant was harvested for determining virus titer through TCID_50_, and the results indicated that PRV titers decreased (Figure 4(b)). According to the IFA assay result, PLP decreased the numbers of infected cells (Figure 4). These results confirmed that PLP inhibited PRV attachment to PK15 cells.

### 3.4. PLP Reduces PRV Penetration into PK15 Cells

For investigating PLP's role in virus penetration into PK15 cells, we infected cells by PRV XJ5 (MOI = 0.1) within DMEM without PLP for a 1 h period at 4°C, and cultured them within 2% DMEM that contained a corresponding concentration of PLP (100, 200, 400, and 600 *μ*g/mL) for a 1 h period under 37°C. After rinsing thrice by citric acid solution and PBS for removing those noninternalized virus particles, cells were maintained in 2% DMEM. At 24 hpi, the western blot, TCID_50,_ and IFA results confirmed that PLP inhibits PRV penetration into PK15 cells dose dependently (Figures 5(a)–5(c)).

### 3.5. The Effect of PLP on Virus Replication

To clarify whether PLP could suppress PRV replication, we incubated PK15 cells by PLP (100, 200, 400, and 600 *μ*g/mL) after 1 h infection by PRV XJ5 (MOI = 0.1) at 37°C. We harvested cells at 4 and 6 hpi to detect PRV gB protein expression levels. The western blot results showed that PRV gB protein expression did not change. In addition, qRT-PCR was carried out to check the change in PRV DNA copy numbers. PLP was found not to affect PRV DNA copy numbers; thus, indicating that PLP did not affect virus replication (Figures 6(a) and 6(b)).

### 3.6. Effect of PLP on Virus Inactivation

PRV XJ5 (MOI = 0.1) were pretreated by PLP (100, 200, 400, and 600 *μ*g/mL), and the pretreatment virus was inoculated to Vero cells to determine viral titers to clarify whether PLP could directly inactivate the virus. The TCID_50_ results showed that the virus titer of the pretreated virus did not change (Figure 7(c)); thus, confirming that PLP cannot directly inactivate the virus.

### 3.7. PLP Reduces Intracellular ROS Levels

PK15 cells were treated as described previously, followed by measurement of ROS contents within PK15 cells by DCFH-DA. The results are observed from Figures 7(a) and 7(b). PLP exposure markedly reduced intracellular ROS levels.

Next, whether N-acetylcysteine (NAC) could inhibit PRV infection by reducing ROS production was explored. We treated PK15 cells by NAC (2, 4, 8, or 10 mM) within DMEM for a 1 h period at 37°C. Subsequently, we inoculated PRV (MOI = 0.1) into cells. After removing NAC-virus supernatant at 1 hpi, we rinsed cells thrice by PBS. After cell incubation by the related NAC doses within 2% DMEM, at 24 hpi, PRV gB protein level decreased dose dependently, suggesting that NAC could inhibit PRV infection by reducing ROS production.

## 4. Discussion

In the past few years, scientists have been working on vaccines and antiviral medicines; however, PR is still a widespread infectious disease in the swine industry [6]. Since the outbreak of PRV variants in 2011, it induced great economic losses in the swine industry [8, 21]. In addition, the report of human infection with PRV has also attracted global attention [9, 22]. Therefore, the development of new anti-PRV medicines is of great significance. Plant polysaccharides are biological macromolecules widely found in the roots, stems, and leaves of plants. Many studies have reported the antiviral effect of plant polysaccharides [23, 24]. *Isatis root* polysaccharide can inhibit H3N2 swine influenza virus *in vivo* and *in vitro* [25]. *Polygonum cillinerve* polysaccharide plays antiviral activity via inhibiting transmissible gastroenteritis virus of swine (TGEV) replication, reducing TGEV-mediated apoptosis and ROS level [26]. Therefore, plant polysaccharides could be a potential source of antiviral medicines.

Recently, researchers mainly focused on polysaccharides in *Plantago asiatica* L seeds. Evidence showed that polysaccharides in *Plantago asiatica* L. seeds could alleviate intestinal barrier injury mediated by nonylphenol [27], resist lipopolysaccharide-mediated liver injury [28], induce dendritic cell maturation [29, 30], and promote lipid metabolism and the development of colonic flora [31]. Compared with the seeds, the whole plants have advantages of lower cost and higher utilization rate. Therefore, the polysaccharide in *Plantago asiatica* L. whole plant was selected to evaluate its antiviral activity in vitro.

According to our results, PLP's antiviral activity in PRV in PK15 cells was evaluated. The results showed that PLP decreased the CPE induced by PRV infection and intracellular viral protein expression dose dependently, which confirmed PLP's antiviral activity in PRV. The first step of PRV infection is that virions bind to heparan sulfate proteoglycans in the extracellular matrix and adsorb to the cell surface. Our study revealed that PLP could reduce PRV attachment in a dose-dependent manner, followed by fusion of viral envelope into the cell membrane, making viral capsid penetrate the cytoplasm [1]. Our study confirmed that PLP decreased PRV penetration into PK15 cells. However, the inhibition of PRV attachment was better than inhibition of PRV penetration. In addition, PLP-pretreated cells could reduce the infectivity of PRV. These results suggested that the antiviral mechanism of PLP may be due to the negative charge on the surface of PLP that interacts with cells' surface protein through electrostatic interaction, thus interfering with the virus attachment to the cells [32, 33]. However, PLP did not affect PRV replication and inactivation.

ROS accounts for the broad definition of oxidizing compounds in organisms, including hydroxyl radical and hydrogen peroxide [34]. Under normal circumstances, intracellular ROS is at a low level but increases rapidly after the virus invades cells, leading to oxidative stress and cell damage [35]. Our results showed that the intracellular ROS level increased after PRV infection in PK15 cells, and the ROS level decreased significantly after PLP treatment, almost reaching the normal level. Related studies have reported that plant polysaccharides have antioxidant and ROS reduction effects [36, 37]. *Ganoderma atrum* polysaccharide can decrease the ROS production in immune organs of immunosuppressive animals and reduce the oxidative damage of immune organs [38]. *Bletilla striata* polysaccharides can reduce angiotensin II-induced oxidative stress and reduce ROS production through NOX4 and TLR2 pathways [39]. In addition, ROS scavenger NAC decreased PRV infection, which confirmed that PLP might reduce ROS to inhibit PRV infection.

Our previous studies have shown that the small molecular medicine EGCG can inhibit PRV and PEDV adsorption, entry, and replication [20, 40]. However, most of the small molecule medicines can only act on a single target. Conversely, plant polysaccharides may be more effective in treating or preventing diseases due to their multicomponent and multifunctional characteristics [41]. Plant polysaccharides are safe with immunoregulation, antioxidation, and antiviral effects and exhibit a wide application prospect in preventing or treating diseases [42].

## 5. Conclusion

In conclusion, we report the inhibitory effect of PLP on PRV infection within PK15 cells. According to this study, PLP plays an anti-PRV role mainly by inhibiting the attachment and penetration of PRV and decreasing ROS. This study can guide the application of PLP, especially for its clinical application as antiviral medicines.

## Figures and Tables

**Figure 1:** PLP inhibited PRV infection within PK15 cells. We pretreated PK15 cells using PLP at diverse doses for a 1 h period prior to PRV XJ5 (MOI = 0.1) infection. We later cultured cells with 2% DMEM that contained PLP for a 24 h period. (a) At 12 and 24 hpi, the changes in cell morphology were observed under a microscope (b). At 24 hpi, *β*-actin and PRV gB protein levels were measured by WB assay. (c) Viral titers were determined by TCID_50._ (d) Internalized virus was evaluated by IFA. The error bars indicated the SD of 3 separate assays. ^∗∗^*P* < 0.01.

**Figure 2:** PLP inhibited PRV infection activity at a different time and different MOI PRV infections. (a) We treated PK15 cells using 0.6 mg/mL PLP for a 1 h period before being infected with PRV XJ5 (MOI = 0.1). *β*-Actin and PRV gB protein levels were assessed by WB assay at 2, 4, 8, 12, and 24 hpi. (b–e) We treated PK15 cells using 400 or 600 *μ*g/mL PLP for a 1 h period, followed by infection using PRV XJ5 at MOI = 0.1, 0.5, 1, or 2, at 24 hpi. *β*-Actin and PRV gB protein expressions were measured using WB. The error bars indicated SD of 3 individual assays. ^∗∗^*P* < 0.01.

**Figure 3:** PLP inhibits PRV attachment and penetration into PK15 cells. (a) We treated PK15 cells by PLP at diverse doses for a 1 h period and then infected by PRV XJ5 (MOI = 0.1) with PLP. At 24 hpi, we conducted WB assay for evaluating *β*-actin and PRV gB protein levels. (b) We infected PK15 cells by PRV XJ5 (MOI = 0.1) for a 1 h period under 4°C with PLP at diverse doses and incubated with different concentrations of PLP at 37°C for a 1 h period prior to removal of PLP DMEM as well as cultivated within PLP-free DMEM. Protein levels of *β*-actin and PRV gB were measured through WB at 24 hpi. (c) We determined virus titers through TCID_50_. (d) We assessed internalized virus through IFA. The error bars indicated SD of 3 individual assays. ^∗^*P* < 0.05, ^∗∗^*P* < 0.01.

**Figure 4:** PLP inhibits PRV attachment onto PK15 cells. (a) We infected PK15 cells by PRV XJ5 (MOI = 0.1) for a 1 h period under 4°C with PLP at diverse doses, followed by removing the PLP DMEM and culturing in PLP-free DMEM. WB assay was conducted to measure the protein levels of *β*-actin and PRV gB at 24 hpi. (b) TCID_50_ was used to detect viral titer. (c) IFA detection of PRV-infected cells. The error bars indicated SD of 3 individual assays. ^∗^*P* < 0.05, ^∗∗^*P* < 0.01.

**Figure 5:** PLP inhibits PRV penetration into PK15 cells. (a) We infected PK15 cells by PRV XJ5 (MOI = 0.1) for a 1 h period at 4°C with PLP, followed by 1 h PLP treatment at diverse doses prior to removing the PLP DMEM and culture in PLP-free DMEM. Protein levels of *β*-actin and PRV gB were measured through WB at 24 hpi. (b) Viral titers were determined through TCID_50_. (c) Internalized virus was evaluated by IFA. The error bars indicated SD of 3 separate assays. ^∗^*P* < 0.05, ^∗∗^*P* < 0.01.

**Figure 6:** We infected PK15 cells using PRV XJ5 (MOI = 0.1) for a 1 h period at 37°C without PLP, followed by incubation using different concentrations of PLP. (a, b) We harvested cells at 4 and 6 hpi for detecting *β*-actin and PRV gB protein expressions through WB. (c, d) qRT-PCR was conducted to quantify copy numbers of viral DNA. The error bars indicated SD of 3 separate assays.

**Figure 7:** PLP reduces intracellular ROS levels. (a, b) We pretreated PK15 cells by PLP at diverse doses for a 1 h period prior to infection by PRV XJ5 (MOI = 0.1), followed by PLP treatment for a 24 h period at diverse doses. Flow cytometry was conducted to measure the total fluorescence intensity of more than 10,000 cells in each sample. (c) We pretreated PK15 cells with different concentrations of NAC (2, 4, 8, or 10 mM). Next, we inoculated PRV (MOI = 0.1) in cells for a 1 h period, followed by incubation using the relevant NAC contents within 2% DMEM. (d) PRV XJ5 (MOI = 0.1) was incubated with PLP (100, 200, 400, and 600 *μ*g/mL) for a 1 h period at 37°C; then, we inoculated the pretreated virus to Vero cell for measuring virus titer through TCID_50_. The error bars indicated the standard deviation from three independent experiments. ^∗∗^*P* < 0.01.

## Data Availability

We have already included the available data in our manuscript.
